This article has been retracted.

# Clinical Effect of Apatinib Mesylate Tablets Combined with Paclitaxel Concurrent Radiotherapy and Chemotherapy in the First-Line Treatment of Locally Advanced Nasopharyngeal Carcinoma

**DOI:** 10.1155/2022/6293816

**Published:** 2022-08-11

**Authors:** Dechao Zhan, Zihong Chen, Donghong Yang, Jiyu Wen, Wanwan Liu

**Affiliations:** Cancer Center, Affiliated Hospital of Guangdong Medical University, Zhanjiang 524000, Guangdong, China

## Abstract

**Objective:**

To explore the clinical efficacy and safety of apatinib combined with paclitaxel in the first-line treatment of locally advanced nasopharyngeal carcinoma.

**Methods:**

From March 2016 to June 2018, 114 patients with locally advanced nasopharyngeal carcinoma who received first-line treatment in our hospital were selected as the patient group, and those who received apatinib combined with paclitaxel concurrent radiotherapy and chemotherapy were selected as the research group (*n* = 54), while those who received paclitaxel concurrent radiotherapy and chemotherapy were selected as the control group (*n* = 60). Sixty healthy individuals in our hospital were recruited in the same period as the healthy group. The clinical effective rate, adverse reactions, 2-year overall survival rate (OS), 2-year progression-free survival rate (PFS), and quality of life were compared between the two groups, and the expression of miR-655 in the serum of each group was tested by RT-qPCR.

**Results:**

The total clinical effective rate of the research group was higher than that of the control group, and the 2-year OS and PFS of the research group were also higher than those of the control group (*P* < 0.05). Both groups of patients could tolerate the treatment, but the incidence of hypertension and proteinuria in the research group was higher than that in the control group (*P* < 0.05). The expression of miR-655 in the serum of patients was lower than that of the healthy group (*P* < 0.05). After treatment, miR-655 in serum increased in both the groups and miR-655 in the research group was higher than that in the control group (*P* < 0.05). The 2-year survival rate of OS and PFS in patients with low expression of miR-655 was significantly lower than that in patients with high expression of miR-655 (*P* < 0.05).

**Conclusion:**

Apatinib combined with paclitaxel concurrent radiotherapy and chemotherapy is effective and well-tolerated in the treatment of locally advanced nasopharyngeal carcinoma, which improves the quality of life of patients and can be popularized in clinical practice. In addition, the increase of miR-655 may be a target for treating nasopharyngeal carcinoma.

## 1. Introduction

Nasopharyngeal carcinoma is an epithelial malignancy, which is prone to local infiltration and early distant metastasis [1]. It is estimated that there are about 130,000 new cases of nasopharyngeal carcinoma in the world in 2018, with the highest incidence in south China, southeast Asia, and North Africa [2]. Because of the deep location of nasopharyngeal carcinoma and the lack of obvious clinical signs in the early stage, more than 70% of the patients were diagnosed as locally advanced at the time of visit, and the prognosis is still poor [3]. At present, concurrent radiotherapy and chemotherapy are often used as the standard treatment strategy for locally advanced nasopharyngeal carcinoma, which can effectively reduce the local recurrence rate and improve the survival rate and local control rate [4]. However, some patients with nasopharyngeal carcinoma will relapse after radiotherapy and chemotherapy [5]. Therefore, finding ways to improve the effectiveness of an antitumor regimen and to prolong the disease-free survival time of patients is a hot spot in clinical research.

Tumor angiogenesis is a necessary step for tumor development and metastasis, and the vascular endothelial growth factor (VEGF) and its receptor (VEGFR) act in this process [6]. Previous studies have found that the VEGF/VEGFR is overexpressed in most NPC patients, which is related to the increased risk of metastasis and the decreased survival time of NPC [7–9]. Therefore, inhibiting the VEGF signaling is considered as one of the effective ways to treat NPC patients. The apatinib is an inhibitor of the VEGFR-2, which can inhibit tumor angiogenesis by selectively binding and inhibiting VEGFR-2, so as to control the tumor development [10]. In 2014, apatinib was approved by China Food and Drug Administration for the treatment of advanced gastric cancer. However, apatinib has not been approved for the treatment of nasopharyngeal carcinoma, and relevant clinical trials are still needed. The microRNA (miR) is a kind of noncoding small RNA, which is widely distributed in animals and plants. By binding to the 3′UTR region of the target gene, it leads to the degradation of mRNA or the inhibition of mRNA translation, thus regulating gene transcription and translation [11, 12]. Through deep understanding of miR, it is found that miR can participate in various tumor development processes and is considered as an important potential target for tumor therapy [13]. MiR-655 is a member of miR, which has been widely considered because its expression is downregulated in many malignant tumors and plays a role in inhibiting tumors [14–16]. However, the role of miR-655 in nasopharyngeal carcinoma is not clear.

This research explored the clinical efficacy and safety of combining apatinib with paclitaxel concurrent chemoradiotherapy in the treatment of locally advanced nasopharyngeal carcinoma [17].

## 2. Materials and Methods

### 2.1. Research Participants

Altogether 114 patients with locally advanced nasopharyngeal carcinoma (stage III, IVa of the seventh edition ofAJCC) who received first-line treatment in our hospital from March 2016 to June 2018 were selected as the patient group, and those who received apatinib combined with paclitaxel concurrent radiotherapy and chemotherapy were selected as the research group (*n* = 54), while those who received paclitaxel concurrent radiotherapy and chemotherapy were selected as the control group (*n* = 60). Inclusion criteria: patients were first diagnosed with nasopharyngeal carcinoma by endoscopic pathological biopsy; the estimated survival time was ≥12 months; the status of the eastern cooperative oncology group (ECOG) was ≤1; Karnofsky (KPS) score was ≥80 points. Exclusion criteria: those with contraindications of radiotherapy; those with distant metastasis; those with contraindications for the use of drugs in this research; those combined with malignant tumors of other systems; those who suffered from mental system diseases; those with dysfunction of important organs such as heart, liver, and kidney; those with incomplete clinical data; due to mental illness or poor compliance, the patient was unable to cooperate with the established treatment plan; those dropped halfway; and pregnant or lactating women. In the same period, 60 healthy individuals in our hospital were recruited as the healthy group, and there were 36 males and 24 females, with an average age of 48.36 ± 5.71 years and an average BMI of 23.91 ± 1.21 kg/m^2^ in the healthy group. There was no statistical difference in the general information between the patient group and the health group. All participants voluntarily signed the informed consent, and this study conformed to the ethics committee.

### 2.2. Therapeutic Method

The control group was treated with paclitaxel concurrent radiotherapy and chemotherapy. The operation was as follows: in the supine position, the patient's neck, nasopharynx, and skull base were irradiated in vitro by MV-X-ray. The total dose of nasopharyngeal irradiation was 66∼74 Gy for 6.5∼7.5 weeks. Patients with lymph node metastasis were administered with 66–74 Gy irradiation. On the 1st, 22nd and 43rd days during radiotherapy, paclitaxel (135-175mg/m^2^) was administered intravenously, for 3 weeks as one chemotherapy cycle, and the patients had undergone 3 cycles of treatment. In the research group, on the basis of the treatment in the control group, at the same time each day, half an hour after a meal, patients were orally administered 500 mg apatinib mesylate tablets (Approval number:H20140103; Jiangsu Hengrui Pharmaceutical Co., Ltd.; 250 mg/s) once daily with concurrent radiation and chemotherapy. Adverse reactions were closely monitored during the use and were adjusted as needed to allow the patient to tolerate the treatment with continuous administration of apartinib mesylate until disease progression or intolerable adverse reactions occurred/disappeared.

### 2.3. Outcome Measures

After the treatment, the clinical curative effect was evaluated according to RECIST1.1, which was divided into complete remission (CR), partial remission (PR), stable disease (SD), and progressive disease (PD). The total effective rate was calculated as total effective rate = (CR + PR)/total cases × 100%.

Two groups of patients were followed up for 2 years by outpatient service, telephone calls and by visiting, and the 2-year overall survival (OS) and the disease progression-free survival (PFS) curves were established. The OS is the time from the start of the treatment to the death or the last follow-up, while PFS is the time from the start of treatment to tumor progression or death.

Adverse reactions of the two groups during treatment were recorded, including the bone marrow suppression, impaired liver and kidney function, dermatitis, diarrhea and vomiting, dry mouth and sore throat, leukopenia, and thrombocytopenia.

The EORTC QLQ-C30 was used to evaluate the quality of life, including body, role, emotion, cognition, and society. The higher score indicated the better quality of life.

### 2.4. RT-qPCR Detection

Before and after treatment, 5 ml of venous blood was collected from the patients in the two groups, while 5 ml of venous blood in the healthy group was collected after entering the group. The samples were sent to the laboratory for centrifugation, and the upper serum was collected and placed for later use. The total RNA was extracted from the serum samples using the TRIzol kit (Invitrogen, USA), and the purity, concentration, and integrity of the extracted total RNA were tested using the ultraviolet spectrophotometer and agarose gel electrophoresis, followed by reverse transcription by using the reverse transcription kit (Invitrogen, USA). The amplification was carried out by using the SYBR_Premix ExTaq II (Takara, China) and the ABI 7500PCR instrument (Applied Biosystems, USA). The amplification system was the SYBR Premix Ex Taq II (2X) (10 *μ*L), the cDNA (2 *μ*L), and the upstream and downstream primers (0.8 *μ*L). Sterile purified water was supplemented to 20 *μ*L, and the amplification conditions were predenatured at 95°C for 30 s, then denatured at 95°C for 5 s, and annealed and extended at 60°C for 30 s, for a total of 40 cycles. Each sample was provided with 3 repeated wells, and the experiment was repeated 3 times. The U6 was applied as the internal reference of the miR, and 2^−△△ct^ was applied to test these data [18].

### 2.5. Statistical Method

The research data were analyzed by using the SPSS 18.0 (EASYBIO), and the pictures were visualized by the GraphPad Prism 7. The counting data were expressed by *n* (%) and compared by the Chi-square test. The measurement data were expressed by (*x*±sd) and compared by the independent sample *t*-test, and the paired *t*-test was applied for intragroup comparison before and after treatment. The Kaplan–Meier method was used to visualize the OS curve for 2 years, and the log-rank test was used to analyze the difference in survival rate between the two groups. *P* < 0.05 represented a statistical difference.

## 3. Results

### 3.1. General Data

There was no significant difference in the general data such as gender, age, BMI index, KPS score, TNM stage, smoking history, and ECOG score between the two groups (*P* > 0.05) (Table 1).

### 3.2. Clinical Efficacy

In the control group, there were 21 cases of CR (35.00%), 18 cases of PR (30.00%), 17 cases of SD (28.33%), and 4 cases of PD (6.67%), with a total effective rate of 65.00%. In the research group, there were 26 cases of CR (48.15%), 19 cases of PR (35.19%), 8 cases of SD (14.81%), and 1 case of PD (1.85%), with a total effective rate of 83.33%. The total effective rate of the research group was higher than that of the control group (*P* < 0.05) (Table 2).

### 3.3. Comparison of OS and PFS in Two Years

During the two-year follow-up, in the research group, 4 cases died and 6 cases experienced disease progression, and in the control group, there were 13 cases and 18 cases who experienced disease progression. The two-year OS (*P*=0.0333, logrank test) and PFS (*P*=0.025, logrank test) of the research group were higher than those of the control group (Figure 1).

### 3.4. Adverse Reaction

During the treatment, no drug allergies occurred in the patients, and the patients tolerated the treatment well. There was no significant difference in the incidence of bone marrow suppression, impaired liver and kidney function, dermatitis, diarrhea and vomiting, and hand-foot syndrome between the two groups during treatment (*P* > 0.05), but the incidence of hypertension and proteinuria in the research group was higher than that in the control group (*P* < 0.05) (Table 3).

### 3.5. Comparison of Quality of Life

The QLQ-C30 showed that there was no significant difference in the scores of QLQ-C30 before treatment between the two groups (*P* > 0.05). After treatment, the scores in the two groups increased significantly, but the scores in the research group were higher than those in the control group (*P* < 0.05) (Figure 2).

### 3.6. Comparison of miR-655 in Serum of Each Group

miR-655 in the serum of the healthy group and the patient group before treatment was tested using the RT-qPCR, and miR-655 in the patient group was significantly lower than that of the healthy group (*P* < 0.05). There was no significant difference between the two groups before treatment (*P* > 0.05). After treatment, miR-655 in both the groups increased significantly, and miR-655 in the research group was higher than that in the control group (*P* < 0.05) (Figure 3).

### 3.7. Relationship of miR-655 with the Prognosis of Patients

According to the median expression of miR-655 in serum before treatment, the patients were divided into the high expression group and low expression group. During the two-year follow-up, in the research group, 5 cases died and 5 cases experienced disease progression; in the control group, there were 12 cases and 19 cases experienced disease progression. The two-year OS and PFS curves showed that the two-year OS of the high expression group was higher than that of the low expression group (*P*=0.024, log-rank test), and the two-year PFS of the high expression group was also higher than that of the low expression group (*P*=0.019, log-rank test) (Figure 4).

## 4. Discussion

At present, concurrent radiotherapy and chemotherapy have become the main choice for nasopharyngeal carcinoma. However, nasopharyngeal carcinoma is prone to recurrence and early metastasis, thus leading to poor prognosis [19]. In recent years, with the clinical application of targeted drugs, there is one or more treatments for cancer patients. In the tumor microenvironment, the growth and metastasis of the cancer cells depend on the angiogenesis of the new tumor, and this process is closely related to the activation of the VEGF signaling pathway [20]. Apatinib is a new type of oral antiangiogenesis agent, and its anticancer effect is by inhibiting the activation of the VEGF pathway, which can inhibit tumor angiogenesis [21]. Previous studies have shown that the apatinib can inhibit the growth of nasopharyngeal carcinoma xenografts [22]. There is also a retrospective study, which shows that apatinib has good efficacy and safety in patients with recurrent and refractory nasopharyngeal carcinoma [23]. However, there is a lack of clinical control studies on the apatinib in the treatment of nasopharyngeal carcinoma. The results of this study showed that the total clinical effective rate of the research group was higher than that of the control group, and the 2-year OS and PFS of the research group were also higher than those of the control group, indicating that paclitaxel concurrent chemoradiotherapy combined with apatinib can improve the therapeutic effect on locally advanced nasopharyngeal carcinoma. As we all know, chemotherapy or radiotherapy will cause a series of side effects, such as oral mucosal disease, pain, fatigue, and dysphagia, which can seriously affect the quality of life of the patients. The occurrence of the adverse reactions in the two groups of patients during treatment was recorded, and both the groups of patients could tolerate the treatment, and only the incidence of hypertension and proteinuria in the research group was higher than that in the control group. With the development of oncology, the survival rate of nasopharyngeal carcinoma patients has been greatly improved, and the high survival rate makes the quality of life high[24]. Therefore, finding ways to prolong the survival time and to ensure the quality of life of patients has become a research hotspot. The quality of life of the patients in the two groups was tested, and the scores of the QLQ-C30 scale in the research group were higher than those in the control group after treatment. This may be because of the better clinical efficacy, which enhances patients' confidence in overcoming diseases and reduces their negative emotions.

MiR has been proved to act as a tumor promoter or inhibitor in the pathogenesis of tumors and is considered as a new target for tumor therapy [25]. miR-655 is a newly reported miR in the recent years, and many research results show that it acts as a tumor suppressor gene in tumors. Studies have found that the miR-655 can inhibit the proliferation and the migration of ovarian cancer cells by targeting the RAB1A [26]. Other studies suggested that low miR-655 correlated with the worse prognosis of esophageal cancer patients, and high miR-655 can inhibit the proliferation and invasion of esophageal cancer cells [27]. However, the role of miR-655 in nasopharyngeal carcinoma is unclear. In this study, miR-655 was low as expressed in the serum of the patients with locally advanced nasopharyngeal carcinoma, and the low expression of miR-655 was related to the worse 2-year OS and PFS of the patients with nasopharyngeal carcinoma, indicating that miR-655 also plays as an anticancer gene in nasopharyngeal carcinoma. Subsequently, this paper also found that miR-655 in both the groups increased significantly after treatment, and miR-655 in the research group was higher than that in the control group. This further indicated that miR-655 was closely related to the patient's disease progression and was expected to be a therapeutic target and an indicator for monitoring the adverse prognosis of nasopharyngeal carcinoma.

There are some shortcomings in this study. Firstly, the small sample size will lead to inevitable selection deviation or measurement deviation, which may weaken the relative reliability of our research results. Secondly, only two years of follow-up were conducted, and the long-term results of the two groups of patients could not be obtained. Finally, this study is a clinical trial, and no basic experiment has been added to analyze the effect of the miR-655 on the growth of nasopharyngeal carcinoma cells. These are expected to be supplemented by more studies in the future.

To sum up, apatinib combined with paclitaxel concurrent radiotherapy and chemotherapy is effective and well-tolerated in the treatment of locally advanced nasopharyngeal carcinoma, which improves the quality of life of patients and can be promoted in clinical practice. In addition, the increase of miR-655 may be a target for treating nasopharyngeal carcinoma.

## Figures and Tables

**Figure 1:** Comparison of the OS and PFS in two years. (a) The OS of the research group was higher than that of the control group in 2 years. (b) The PFS of the research group was higher than that of the control group in 2 years.

**Figure 2:** Comparison of the QLQ-C30 scores. Comparison of (a) body scores, (b) role scores, (c) emotional scores, (d) cognitive scores, and (e) social scores between the two groups before and after treatment. Note: ^*∗*^ represents the comparison before and after treatment, *P* < 0.05; ^#^ means compared with the control group at the same time, *P* < 0.05.

**Figure 3:** Comparison of miR-655 in serum of each group. (a) MiR-655 in the patient group was significantly lower than that of the healthy group. (b) After treatment, miR-655 in both groups increased significantly, and miR-655 in the research group was higher than that in the control group. Note: & means compared with the healthy group, *P* < 0.05; ^*∗*^ means the comparison before and after treatment, *P* < 0.05; ^#^ means compared with the control group at the same time, *P* < 0.05.

**Figure 4:** Relationship of miR-655 with the prognosis of patients. (a) OS of the high expression group was higher than that of the low expression group in 2 years. (b) PFS of the high expression group was higher than that of the low expression group in 2 years.

**Table 1:** Comparison of the general data (*n* (%), (*x* ± sd).

Group	Control group (*n* = 60)	Research group (*n* = 54)	*χ* ^2^/*t*	*P*
Gender			0.199	0.656
Male	38 (63.33)	32 (59.263)		
Female	22 (36.673)	22 (40.743)		
Age (years)	48.48 ± 7.25	47.26 ± 6.89	0.918	0.360
BMI (kg/m^2^)	23.75 ± 1.48	24.05 ± 1.38	1.116	0.267
KPS score	86.45 ± 4.64	87.55 ± 4.34	1.303	0.195
TNM staging			0.958	0.619
III	44 (73.33)	36 (66.67)		
IVa	11 (18.33)	14 (25.93)		
IVb	5 (8.33)	4 (7.41)		
History of smoking			0.594	0.441
Yes	29 (48.33)	30 (55.56)		
No	31 (51.67)	24 (44.44)		
ECOG score			0.691	0.406
0	21 (35.00)	23 (42.59)		
1	39 (65.00)	31 (57.41)		

**Table 2:** Comparison of clinical efficacy (*n* (%)).

Group	Control group (*n* = 60)	Research group (*n* = 54)	*χ* ^2^	*P*
CR	21 (35.00)	26 (48.15)		
PR	18 (30.00)	19 (35.19)		
SD	17 (28.33)	8 (14.81)		
PD	4 (6.67)	1 (1.85)		
Total effective rate	39 (65.00)	45 (83.33)	4.926	0.026

**Table 3:** Comparison of toxic and side effects (n (%)).

Group	Control group (*n* = 60)	Research group (*n* = 54)	*χ*2	*P*
Bone marrow suppression	12 (20.00）	17 (34.18)	1.975	0.160
Impaired liver and kidney function	7 (11.67）	11 (20.37)	1.619	0.203
Dermatitis	10 (16.67）	17 (34.18)	3.451	0.063
Diarrhea and vomiting	19 (31.67）	22 (40.74)	1.016	0.313
High blood pressure	12 (20.00）	20 (37.04)	4.086	0.043
Proteinuria	9 (15.00）	17 (31.48)	4.385	0.036
Hand-foot syndrome	8 (13.33）	14 (25.93)	1.913	0.089

## Data Availability

The data used and/or analyzed during the current study are available from the corresponding author.
